The article "Artificial intelligence in psychodermatology: A brief report of applications and impact in clinical practice" was published in 2024. Journal: Skin Res Technol.

# Artificial intelligence in psychodermatology: A brief report of applications and impact in clinical practice

**DOI:** 10.1111/srt.70044

**Published:** 2024-08-29

**Authors:** Isabella J. Tan, Olivia M. Katamanin, Rachel K. Greene, Mohammad Jafferany

**Affiliations:** ^1^ Robert Wood Johnson Medical School Rutgers, the State University of New Jersey Piscataway New Jersey USA; ^2^ Chicago Medical School Rosalind Franklin University North Chicago Illinois USA; ^3^ University of California San Diego San Diego California USA; ^4^ Department of Psychiatry and Behavioral Sciences Central Michigan University College of Medicine Mount Pleasant Michigan USA

**Keywords:** artificial intelligence, dermatology, diagnostic accuracy, healthcare innovation, psychodermatology, treatment optimization

## Abstract

**Background:**

This report evaluates the potential of artificial intelligence (AI) in psychodermatology, emphasizing its ability to enhance diagnostic accuracy, treatment efficacy, and personalized care. Psychodermatology, which explores the connection between mental health and skin disorders, stands to benefit from AI's advanced data analysis and pattern recognition capabilities.

**Materials and methods:**

A literature search was conducted on PubMed and Google Scholar, spanning from 2004 to 2024, following PRISMA guidelines. Studies included demonstrated AI's effectiveness in predicting treatment outcomes for body dysmorphic disorder, identifying biomarkers in psoriasis and anxiety disorders, and refining therapeutic strategies.

**Results:**

The review identified several studies highlighting AI's role in improving treatment outcomes and diagnostic accuracy in psychodermatology. AI was effective in predicting outcomes for body dysmorphic disorder and identifying biomarkers related to psoriasis and anxiety disorders. However, challenges such as limited dermatologist knowledge, integration difficulties, and ethical concerns regarding patient privacy were noted.

**Conclusion:**

AI holds significant promise for advancing psychodermatology by improving diagnostic precision, treatment effectiveness, and personalized care. Nonetheless, realizing this potential requires large‐scale clinical validation, enhanced dataset diversity, and robust ethical frameworks. Future research should focus on these areas, with interdisciplinary collaboration essential for overcoming current challenges and optimizing patient care in psychodermatology.

## 1 INTRODUCTION

Psychodermatology explores the relationship between mental health and skin disorders, recognizing how psychological factors can significantly influence skin conditions.^1^ Concurrently, artificial intelligence (AI) represents a transformative technology in healthcare, leveraging computational systems to replicate human cognitive functions.^2^ In dermatology, AI has reshaped diagnostic approaches and treatment strategies, showcasing its potential to improve precision and efficiency. The integration of AI into psychodermatology holds promise for advancing diagnostics and therapeutic interventions, aiming to optimize patient care outcomes by leveraging AI's capabilities in data analysis and pattern recognition.^3^ Understanding AI's implications in psychodermatology necessitates evaluating its potential to enhance diagnostic accuracy and treatment efficacy while addressing ethical considerations and the need for robust validation frameworks. This report reviews the existing literature to assess AI's impact on psychodermatology, synthesizing evidence to inform clinical practice and guide future research directions.

The article "Artificial intelligence in psychodermatology: A brief report of applications and impact in clinical practice" was published in 2024. Journal: Skin Res Technol.

## 2 MATERIALS AND METHODS

This report was conducted in accordance with Preferred Reporting Items for Systematic Reviews and Meta‐Analysis (PRISMA) guidelines^4^ and registered with PROSPERO (568298). To assess the risk of bias, we utilized the Critical Appraisal Skills Program (CASP) tool categorizing the risk as high (0–3), moderate (4–6), or low (7+). A comprehensive search of PubMed and Google Scholar (2004–2024) was performed using the search thread: “artificial intelligence” AND “psychodermatology” OR “machine learning” AND “skin disorders.” After duplicate removal, titles and abstracts were screened for eligibility, with full‐text evaluation used when necessary. Inclusion criteria focused on studies applying AI to psychodermatological conditions, involving human subjects, and published in English within the last 20 years. Exclusion criteria included non‐English publications, studies outside the timeframe, and those not focused on AI in psychodermatology. Data were extracted, categorized, and synthesized to derive insights into AI's impact and application in the field.

## 3 RESULTS

Study selection adhered to predefined inclusion and exclusion criteria. One hundred and seventy‐eight studies were initially identified on PubMed and Google Scholar. Subsequent primary and secondary screenings led to the inclusion of three studies (Figure 1). These consisted of one qualitative study, one randomized controlled trial, and one systematic review. Characteristics of the included studies are presented in Table 1. Risk of bias assessment is depicted in Table 2.^5^

**FIGURE 1:** PRISMA flow diagram depicting study selection process.

**TABLE 1:** Study characteristics.

Study characteristics					Methods	Results	AI techniques (algorithms, image analysis)	Impact of AI on psychodermatology
Author	Year	Study design	Patients (*n*)	Control (*n*)				
Curtiss, et al.^8^	2023	Clinical Trial	97	N/A	‐ 97 BDD patients received escitalopram for 14 weeks. ‐ Used 10‐fold cross‐validation support vector machine (SVM) to predict BDD treatment outcomes: partial remission, full remission, response. ‐ Baseline self‐reporting questionnaire and clinical interview data were used for machine learning. ‐ In phase II, responders to the initial treatment were randomly assigned to either continue with 6 months of escitalopram or receive a placebo pill.	‐ 72% of participants achieved response, 51% partial remission, 20% full remission.	Algorithms	‐ Machine learning predicts BDD treatment outcomes, guiding personalized pharmacotherapy strategies. ‐ Identifies psychopathology and hopelessness as predictive factors for treatment outcomes.
Flygare, et al.^6^	2020	RCT	47	47	‐ Random forests machine learning approach used for outcome prediction. ‐ Logistic regression models compared to random forests for outcome prediction of BDD remission.	‐ Random forests predicted BDD remission with 78% accuracy at post‐treatment. ‐ Machine learning models identified key predictors like depressive symptoms, working alliance, initial severity of BDD and treatment credibility	Algorithms	‐ Machine learning predicts BDD remission with key predictors like depressive symptoms. ‐ Random forests detect remitters accurately post‐treatment, guiding personalized care
Liu et al.^7^	2024	Systematic Review	N/A	N/A	‐ Machine learning algorithms for hub gene screening and diagnostic genes.	‐ Identified key hub genes related to psoriasis autophagy and immune regulation. ‐ Used machine learning algorithms to identify 13 potential psoriasis samples.	Algorithms	‐ Machine learning identifies diagnostic genes related to psoriasis and anxiety disorders. ‐ Biomarkers aid disease prediction and personalized treatment development.

Abbreviations: BDD, body dysmorphic disorder; RCT, randomized control trial.

The article "Artificial intelligence in psychodermatology: A brief report of applications and impact in clinical practice" was published in 2024. Journal: Skin Res Technol.

**TABLE 2:** Risk of bias.

Study number	Study ID	ROB
1	Curtiss et al.	7
2	Flygare et al.	9
3	Liu et al.	9

Abbreviation: ROB, risk of bias.

AI shows promise in psychodermatology, particularly through telehealth. Flygare et al. conducted an RCT with 94 body dysmorphic disorder (BDD) patients randomized to internet‐delivered cognitive behavioral therapy (ICBT) or online supportive therapy for 12 weeks.^6^ Machine learning algorithms, specifically random forests, predicted BDD remission with 78% accuracy.^6^ At the 3‐month follow‐up, 42% were in remission, with the model identifying 68% correctly; at 12 months, 47% were in remission with 66% accuracy; and at 24 months, 60% were in remission with 61% accuracy.^6^ Logistic regression models did not consistently predict remission, highlighting the potential of machine learning for personalized BDD treatment, with machine learning algorithms predicting remission based on key predictors such as depressive symptoms.

Liu et al. explored the impact of psychological stress on skin health by studying individuals with psoriasis, major depressive disorder (MDD) with anxiety, and healthy controls.^7^ Using five machine learning algorithms, the study identified four biomarkers for disease prediction from 16 candidate genes in the gene expression omnibus (GEO) database.^7^ ROC curve analysis showed these biomarkers' predictive capability in both training and validation datasets. The study revealed a potential link between anxiety disorders and increased autophagy, immune dysregulation, and inflammation.^7^ Single‐cell RNA sequencing highlighted the role of the CASP7 gene in psoriasis, suggesting it affects T cell development and immune regulation.^7^ These findings indicate that anxiety may influence skin inflammation and suggest potential biomarkers for predicting and personalizing treatment for both anxiety and psoriasis.

Curtiss et al. used machine learning to predict treatment outcomes for BDD in 97 patients treated with escitalopram for up to 14 weeks.^8^ Support vector machine (SVM) models with 10‐fold cross‐validation achieved AUCs of 0.77 (sensitivity = 0.77 and specificity = 0.63) for treatment response, 0.75 (sensitivity = 0.67 and specificity = 0.73) for partial remission, and 0.79 (sensitivity = 0.70 and specificity = 0.79) for full remission.^8^ Key predictors of better treatment outcomes included lower dermatology life quality index (DLQI) scores and reduced hopelessness, while demographic variables were less predictive.^8^ This study demonstrates that machine learning may have a role in predicting pharmacotherapy outcomes for BDD, supporting the development of personalized treatment plans and aligning with precision medicine in psychiatry and psychodermatology.

## 4 DISCUSSION

AI shows strong potential to enhance diagnostic accuracy, treatment effectiveness, and patient outcomes in psychodermatology. AI‐driven algorithms enable more precise and individualized care by improving screening, diagnosis, and treatment. For example, Flygare et al.’s machine learning models effectively predict body dysmorphic disorder outcomes by identifying key factors like reduced depression severity and improved quality of life.

The real‐world efficacy of AI in psychodermatology requires further validation. Only 13.75% of dermatologists possess a thorough understanding of psychocutaneous disorders.^9^ Challenges such as consultation time, cost, and AI training must be addressed. Concurrently, AI's generalizability is uncertain, and integration is hindered by interoperability issues, provider resistance, and financial constraints.

The article "Artificial intelligence in psychodermatology: A brief report of applications and impact in clinical practice" was published in 2024. Journal: Skin Res Technol.

Policy development for AI in psychodermatology must address ethical concerns such as patient privacy and algorithm transparency, while adjunctively addressing financial barriers.^3^ Policies should support both the necessary technological infrastructure and the training of healthcare providers to ensure equitable access and effective use of AI.

Current impediments in AI for psychodermatology include data diversity and quality issues, integration challenges, ethical concerns, and cost barriers. AI datasets often lack diversity, leading to biased outcomes and limited generalizability. For instance, AI has been shown to inadvertently perpetuate discriminatory practices, recommending less follow‐up for African‐American patients compared to Caucasian patients with similar needs, when healthcare costs are used as a proxy for care.^10^ Addressing these issues requires standard guidelines and regulatory oversight.^10^ Additionally, AI integration demands significant training and support, while provider reluctance and financial constraints hinder widespread adoption. Ethical concerns about patient privacy and algorithmic transparency also complicate AI's clinical implementation.

## 5 LIMITATIONS

This report is limited by the scarcity of studies specifically exploring AI in psychodermatology, with only three studies meeting the inclusion criteria. The heterogeneity of these studies, along with potential biases in the datasets used, limits the generalizability and robustness of the findings.

## 6 CONCLUSION

The present report highlights AI's potential to enhance psychodermatological practice by improving diagnostic accuracy, treatment efficacy, and personalized care. However, challenges such as limited dermatologist knowledge, interoperability issues, and ethical concerns including patient privacy and algorithm transparency hinder AI's clinical integration. Large‐scale trials with validation studies, diverse datasets, and policies to support equitable AI use, emphasizing interdisciplinary collaboration to advance patient care are required. Future research should focus on dataset quality and diversity, refinement of AI algorithms, and addressing ethical and cost challenges. Policies should promote equitable AI access and ensure adequate training for healthcare providers. As AI advances, dermatologists must understand its principles and limitations to optimize psychodermatology and improve patient outcomes through personalized care.

The article "Artificial intelligence in psychodermatology: A brief report of applications and impact in clinical practice" was published in 2024. Journal: Skin Res Technol.

## CONFLICT OF INTEREST STATEMENT

None reported.

## Data Availability

The data that support the findings of this study are available from the corresponding author upon reasonable request.
